# Why do Chinese enterprises make imitative innovation?—An empirical explanation based on government subsidies

**DOI:** 10.3389/fpsyg.2022.802703

**Published:** 2022-09-12

**Authors:** Feifei Song, Changheng Zhao

**Affiliations:** ^1^School of Finance and Public Administration, Hubei University of Economics, Wuhan, China; ^2^School of Economics, Lanzhou University, Lanzhou, China

**Keywords:** government subsidies, imitative innovation, independent innovation, enterprise performance, enterprise innovation

## Abstract

The previous literature analyzed the widespread imitative innovation of Chinese enterprises from various perspectives, including enterprises' rational choice of cost-gain, property rights system, human capital and policy environment. However, this paper provides a brand-new perspective on government subsidies for the reasons behind the imitative innovation of enterprises. According to the statistics from Chinese enterprise-labor matching, we found that government subsidies stimulated enterprises to make “imitative innovation” through patent purchase rather than independent R&D. Government subsidies were used for low-risk “imitative innovation” because of enterprises' rent-seeking behavior, low R&D ability and the review of government subsidy projects. Based on the above conclusions, this paper suggests that the government should reduce or withdraw its intervention in enterprise innovation and implement the post-subsidy and post-evaluation mechanism for government-subsidized programs.

## Introduction

Schumpeter (1991) divided technological innovation into three categories: independent, imitative, and cooperative. Innovation is the transformation of knowledge into economic activities (Tang, 2006). As one of the important factors for improving productivity, independent innovation plays an important role in economic development. However, the enterprises may be less motivated to conduct independent innovation activities because of high risk and income uncertainty.

In China, it is a consensus that innovation can drive economic development, especially enterprises' development. Innovation always serves the development of industry (Taylor, 1993). However, what surprised us is that innovation returns are getting lower. The reason is that China has followed the path of imitative innovation over the past 30 years; that is, China achieves technological progress through the introduction and purchase of technology. There is no doubt that imitative innovation helps China make many innovative achievements in the early stage of enterprise of development. However, with the increasing market demand for innovation, independent innovation, especially the establishment of independent brands, standards, technology and original R&D, becomes particularly important for economic development. Empirical evidence shows that imitative innovation can help latecomer countries to catch up with developed countries in the short-term effects, but it is not conducive to long-term economic growth. Only with independent innovation can long-term economic growth be realized (Aghion et al., 2001). And, creative imitation can improve financial performance (Lee and Zhou, 2012). However, China still has a long way to go before realizing independent innovation.

Scholars have studied why it is difficult for China to make independent innovations. The reasons include enterprises' rational choice of cost-gain, property rights system, culture, human capital, and government subsidies. Two aspects of induction and extrusion effects on enterprise R&D were explored regarding the government subsidies. However, the above explanations, especially the government subsidies, cannot effectively explain why the Chinese government ranks at the top of the world in total R&D investment but lags in innovation capacity. Furthermore, the induction effect and extrusion effect on enterprise R&D only point out that government subsidies can encourage enterprises to increase or decrease R&D expenditure but do not fundamentally explain why enterprise innovation behaviors change, especially the change in enterprise innovation mode selection. China's current incentive system may not be enough to stimulate independent research and development of enterprises (Dai, 2010).

Based on this, this paper will focus on the impacts of government subsidies on enterprise innovation behaviors and analyze why the enterprises mainly adopt imitative innovation. This paper divides enterprise innovation into two types- “independent innovation” and “imitative innovation,” and then analyzes government subsidies will affect which type of innovation. In this study, “independent innovation” means the enterprise's technological progress created from R&D investment, and “imitative innovation” means the technological introduction from other countries. The connotations of “independent innovation” and “imitative innovation” will be further developed in detail. “Independent innovation” includes the total number of patents granted, the number of domestic patents granted, and the number of foreign patents granted, while “imitative innovation” is defined as the total number of patents introduced, the number of domestic patents introduced and the number of foreign patents introduced. The empirical tests will be conducted on whether the government subsidies can promote the imitative innovation of enterprises, and the influence mechanism of government subsidies on imitative innovation will be analyzed. Given this, the in-depth analysis of enterprise innovation behavior should be based on the comprehensive empirical observations of a large number of microscopic data, so this paper will adopt the statistics of Chinese enterprise-labor matching to verify the above issues.

## Literature review

The existing literature explores the reasons behind enterprise imitative innovation. It is believed that the factors for enterprise imitative innovation include the following aspects:

First, innovation is generally regarded as the field of producers (Gambardella et al., 2017) it comes from the enterprise s' rational choice of cost gain. Romer (1990) noted that the non-competition nature of the technology allows a manufacturer to use technology without preventing other manufacturers from using it simultaneously, so the cost of technology imitation can even be as low as zero. Compared with independent innovation requiring substantial human resources, material resources and financial resources, imitative innovation costs a little and can maximize the income with a fixed cost, so enterprises prefer imitative innovation (Aghion et al., 2001; König et al., 2016). Further, at the national level, developing countries can absorb knowledge spillover and achieve endogenous growth through imitation at a low cost in the short term (Barro, 1997). Characterized by low cost and low risk, imitative innovation becomes the best choice for technological progress in developing countries to obtain the existing technologies of developed countries (Vandenbussche and Aghion, 2006) to narrow the economic gap with developed countries.

Second, the system is also an important factor. The change in the intellectual property system in developing countries may hardly obtain bottom-up support, which hinders the innovation-driven development of enterprises. In terms of the imitative innovation behaviors of Chinese enterprises, Zheng and Wang (2012) noted that an imperfect institutional environment would undermine intellectual property protection, so enterprises will follow other innovators and adopt imitative innovation strategies. Besides, a weak legal environment and imperfect property rights system will lead to partial imitative innovation behaviors (Lee and Zhou, 2012). The lack of intellectual property protection will hinder innovation protection rather than bring about imitative innovation behaviors (Taylor, 1993; Yang and Maskus, 2001). Business models under specific systems can also stimulate innovation (Lee and Shin, 2018).

The third factor is human capital. According to Datta and Mohtadi (2006), the transformation from imitation to independent innovation in developing countries is restricted by human capital. It can be said that human capital determines whether an enterprise chooses independent innovation or imitative innovation (Yang et al., 2014). The lack of entrepreneurship, especially entrepreneurial innovation, largely handicaps the improvement of enterprises' technological and innovative ability (Cheng and Song, 2016; Emami and Dimov, 2016; Jahanshahi and Brem, 2018). Moreover, entrepreneurs' original innovation path, especially insufficient R&D investment, determine that enterprises may rely on imitation to improve their technical level (Tang, 2014; Cheng et al., 2016).

Fourth, culture also has influenced. Culture, as a factor underpinning enterprise behavior, has an important influence on enterprise innovation. Enterprises are essentially culturally driven when they need to choose whether to pioneer in innovation or imitative innovation (Hartmann, 2006). Gallagher and Worrell (2008) pointed out that enterprises with a market culture (strong market competition) generally attach great importance to R&D output and market demand, so they may choose an imitative innovation path which requires less time. Similarly, Zhang and Chen (2014) believed that enterprises with hierarchical cultures attach great importance to stability and undisruptive innovation, so they may choose an imitative innovation method with less innovation investment and low innovation risk.

Fifth, government subsidies are also a key. Most scholars explain the influence of government subsidies on enterprise R&D from the two aspects: “induction effect” and “extrusion effect.” Scholars for the “induction effect” view believe that as market failure brings a reduced risk and preference for enterprise R&D investment, the government can stimulate the enterprises to increase R&D expenditure through government subsidies and improve innovation performance (Arrow, 1972; Czarnitzki and Hussinger, 2004; Mateut, 2017). However, there is evidence on whether such improved innovation performance is an independent one or not. Scholars for the “extrusion effect” believe that government subsidies will have an extrusion effect on the R&D investment activities of enterprises, that is, enterprises may reduce their R&D investment and output of independent R&D activities (Link, 1982; Wallsten, 2000; Cheng et al., 2019; Kuehnl et al., 2019). However, the use of extrernal funding increases with firm's innovation effort (Bartoloni, 2013).

However, based on the above explanations, the literature fails to explain under what conditions enterprises choose imitative innovation and why enterprises choose imitative innovation? In particular, the government subsidies cannot fundamentally explain the change in enterprise innovation behavior, especially the change in enterprise innovation mode selection. Therefore, this paper innovatively analyzes the reasons behind enterprise imitative innovation based on government subsidies and then explores the internal influence mechanism of the reasons. Based on the microdata of enterprise-labor matching, this paper will discuss the empirical impact of government subsidies on two different innovation types of enterprises, analyze the heterotrophic influences of different kinds of government subsidies, and put forward policy recommendations to avoid the imitative innovation of Chinese enterprises in the future.

Recently, innovation has attracted extensive attention in the economic field, and many scholars focus on this important issue. Kovalenkov and Vives (2008) captured the relationship between competition and innovation. She et al. (2017) discussed the relationship between financial structure and innovation and found that financial structure affects innovative investment. Nie et al. (2017) examined the effects of switching costs on innovative investment. Nie and Yang (2020) characterized the innovation under capacity constraints and showed that rare resource deters innovative investment. All the existed literature about innovation concludes underinvestment phenomena in innovation. To stimulate innovation, governmental intervention seems to be an efficient tool. Acemoglu and Ufuk (2012) showed that intellectual property rights policy improves innovation. The governmental subsidy is regarded as another tool to stimulate innovation. In theory, Wang et al. (2018) argued that subsidy for insurance improves green innovation. Cheng et al. (2019) proved that governmental subsidy improves the environmental effects of the supply chains of the firm. Huang et al. (2019) argued that innovation subsidy improves production quality.

Much empirical evidence also identifies that subsidy improves innovation. Leibowicz (2018) found that subsidies improve innovation with stronger spillovers and moderately costly research and development to a great degree. Marino et al. (2016) identified the crowding out effects of public research and development subsidies on private firms. Buchmann and Micha (2019) checked the German biotech industry and found that subsidy increases the number of patents. Interestingly, based on the data from Slovakia, Kuehnl et al. (2019) found that innovation subsidy has significantly positive effects on labor productivity, whereas these effects disappear after 1 year. Zhang and Guan (2018) also identified time-varying phenomena about innovation subsidies. Szücs (2018) checked the stimulating impact of innovation subsidy on innovation cooperation between firms and universities. In summary, both theoretical and empirical conclusions show that subsidy improves innovation. Many papers focus on the subsidizing mechanism to achieve the best efficiency. Chen et al. (2017) analyzed the subsidy in the agricultural sector. Arkolakis et al. (2018) addressed innovation under global economy. Nie et al. (2017) compared input subsidy with output one and found that output subsidy plays an advantage based on consumers. Wang et al. (2018) proposed insurance subsidies to improve innovation. Recently, Yang et al. (2014) considered governmental subsidy in renewable energy projects and showed that governmental subsidy enhances the success of renewable energy development. Recently compared input with output subsidy under uncertainty and concluded that input subsidy reduces risk. Although the subsidy mechanism is extensively investigated, no research focuses on the subsidy mechanism under the asymmetric situation.

Likewise, Nie et al. (2020) also tried to investigate the subsidized innovation efficiency under the prism of game theory. They found the U-shaped relationship between subsidized firms' innovations and product sustainability. Also, they demonstrated that those firms denoted with high subsidize firms had more output compared with low subsidize firms. Finally, they concluded that bilateral subsidy brings more innovations than unilateral subsidy. Similarly, Nie et al. (2020) also tried to investigate the innovation strategies concerned public and private firms to capture the welfare effect of public ownership. They found that private firms responded more to research and development activities than public firms. Also, they pointed out the significant loss in profit due to an increase in total productivity via the degree of public ownership. According to the policy suggestions, the mixed economy can significantly boost the shortcomings mentioned.

## Data sources and sample selection

### Data sources and samples

Wuhan University, the author's alma mater, the University of Hong Kong University of Science and Technology, Tsinghua University and the Chinese Academy of Social Sciences carried out a large-scale first-hand enterprise survey to achieve academic research. This survey was originally launched in 2012. After 2 years of questionnaire design, trial survey, communication and coordination, and 5 field simulation surveys and summary on trial and errors from October 2014 to May 2015, the field survey was completed in May-August 2015 and May-August 2016, respectively.

To ensure sample heterogeneity and representativeness, this research selected Guangdong Province's largest economic aggregate, manufacturing scale, and significant regional economic development gap as the survey region. Hubei Province, with the economic aggregate at the medium level in China, was selected as the control region. The survey adopted a strict random hierarchical sampling method compared with the existing data. Specifically, according to the principle of isometric sampling, 13 prefecture-level cities were randomly selected from each province, and 19 districts (counties) under the jurisdiction of 13 prefecture-level cities were selected as the final survey units. The enterprise samples were selected according to the number of employees in the enterprise list of the third economic census by weighted sampling, and the employee samples were selected based on 30% of the middle and senior enterprise managers and 70% of the front-line employees in the employee list of the survey enterprises by stratified random sampling. This time, the probability distribution based on a strict random hierarchical sampling method was consistent with the real distribution of enterprises and employees.

From the perspective of enterprise information, entrepreneurs' personal information and employee information, the survey was the first large sampling survey on enterprises in large developing economies, except for small Nordic economies such as Denmark and Norway. The survey fully collected enterprise information, such as innovation performance, scale, Age of enterprise, capital, ownership type, export or not, and various types of government subsidies enjoyed by the enterprises. Most importantly, the data included enterprise imitative innovation and independent innovation and other indexes, thus providing complete data for studying why Chinese enterprises form imitative innovation.

### Test model

According to the research needs, this paper built the following model:


(1) $$\begin{array}{r} \text{lninnovation}=\alpha 0+\alpha +\alpha \text{2Cij}+\text{Ai}+\text{Ij}+\mu_{IJ} \end{array}$$

Where innovation was the innovative performance of the *j*th enterprise in the *i*th region, subisidy_ij_ referred to the government subsidies accepted by the *j*th enterprise in the *i*th region, C_ij_ was the control variables; I_j_ meant the fixed effect of region and industry, and U_ij_ was the random disturbance term. Other variables in the model were set as their natural logarithm except for the dummy variables. The variables in the model were defined as follows:

#### Dependent variable

The dependent variable was the innovation performance of enterprises. Since the innovative performance was mainly about the transformation or industrialization of innovation achievements, the sales of new products were used as the proxy variable of enterprise innovation performance according to OECD's method 1997 for measuring innovation performance. This indicator reflected the performance after the industrialization of innovation achievements and the applied performance (Chen and Chen, 2006). Crepon et al. (1998) and Pellegrino et al. (2012) have studied the innovative ability based on the development or sales of new products of enterprises. Therefore, the sales of new products that reflect process and product innovation were suitable for this paper.

#### Independent variables

Government subsidies belong to independent variables. It is generally believed that the policy tools for the Chinese government to intervene in enterprise innovation include various science and technology plans, technology innovation funds, fiscal and financial policies, etc. The government subsidies in this paper were all directly related to technologies. Therefore, according to the research needs, the total government subsidies, whether to enjoy government subsidies and other variables were adopted, and the government subsidies were classified to verify the effect of government subsidies on enterprise innovation.

Imitative innovation is also in this category. The key to independent innovation lies in the emphasis on enterprise acquiring technology from other countries or direct purchase or introducing domestic and foreign patents. Therefore, this paper selected the total number of patents introduced and the number of domestic and foreign patents introduced in 2015 to analyze the “imitative innovation.”

Independent innovation is another independent variable. According to the definition given in the “*Statistics on the Independent Innovation of Large and Medium-sized Industrial Enterprises*” compiled by the National Bureau of Statistics, the independent innovation of industrial enterprises refers to the research and experimental development (hereinafter referred to as R&D) activities as well as the patents and other innovation output brought about by the industrial enterprises. This paper adopted the total number of patents granted, the number of domestic patents granted, and foreign patents granted in 2015 as proxy variables for independent innovation.

#### Control variables

According to the research needs, the control variables selected in this paper included: R&D investment used by Liu and Liu (2022), entrepreneurs' education level, Age of enterprise used by Zhang et al. (2021), and scale used by Panfiluk (2021), whether to export, ownership type, etc. Given the differences in the innovation ability in different industries and regions, the model has also controlled the fixed effects of industry and region.

To sum up, the descriptive statistics of the main variables of this paper are shown in Table 1.

**Table 1:** Descriptive statistics.

**Variable name**	**Statistical definition**	**Obs**.	**Mean**	**Std. Dev**.	**Min**	**Max**
Sales of new products	Sales of new products of enterprises in 2015 (10,000 yuan)	1,009	156581.400	4722708	0	1.50E+08
Total government subsidies	Total government subsidies enjoyed by enterprises in 2015 (10,000 yuan)	1,116	41.931	401.761	0	12,295
Whether to enjoy government subsidies?	Whether the enterprises enjoyed government subsidies in 2015? (0-1)	1,117	0.234	0.423	0	1
Environmental subsidies	Total environmental subsidies enjoyed by enterprises in 2015 (10,000 yuan)	1,102	4.521	71.979	0	1,875
High-tech subsidies	Total high-tech subsidies enjoyed by enterprises in 2015 (10,000 yuan)	1,100	14.727	124.267	0	3,120
Technical innovation funds	Total technical innovation funds obtained by enterprises in 2015 (10,000 yuan)	969	4.605	65.783	0	1520.5
Total number of patents granted	Number of patents granted in 2015 (pcs.)	1,057	10.574	106.951	0	2,934
Number of domestic patents granted	Number of domestic patents granted in 2015 (pcs.)	1,085	9.790	85.277	0	2178.333
Number of foreign patents granted	Number of foreign patents granted in 2015 (pcs.)	1,059	1.403	25.759	0	755.667
Total number of patents introduced	Number of patents introduced in 2015 (pcs.)	1,092	0.430	6.844	0	212
Number of domestic patents introduced	Number of domestic patents introduced in 2015 (pcs.)	1,093	0.188	1.972	0	40
Number of foreign patents introduced	Number of foreign patents introduced in 2015 (pcs.)	1,095	0.048	0.796	0	20
R&D investment	Total R&D expenditure in 2015 (10,000 yuan)	809	1828.947	11179.490	0	216,523
Age of enterprise	Years of enterprise establishment (years)	1,086	12.612	7.535	3	62
Scale	Enterprise workforce in 2015 (person)	1,118	1.534	0.751	1	3
Export or not	Whether the enterprises exported in 2015 (0-1)	1,116	0.424	0.494	0	1
Entrepreneurs' education level	Years of entrepreneurs' education (years)	1,186	14.348	3.085	0	22
Private enterprises	Whether the enterprises were private holding enterprises in 2015	734	2	0	2	2
State-owned enterprises	Whether the enterprises were state holding enterprises in 2015	87	1	0	1	1
Foreign enterprises in Hong Kong, Macao and Taiwan	Whether the enterprises were foreign enterprises in Hong Kong, Macao and Taiwan in 2015	184	3	0	3	3
Foreign enterprises in non-Hong Kong, Macao and Taiwan	Whether the enterprises were foreign enterprises in non-Hong Kong, Macao and Taiwan in 2015	109	4	0	4	4

## Empirical test results and analysis

### Basic regression results

Firstly, this paper discussed whether government subsidies could promote enterprise innovation. Under the premise of fully controlling the enterprise, industry, region and other factors, this paper measured the empirical impact of total government subsidies, whether to enjoy government subsidies and other variables on the innovative performance of enterprises. The statistical results are shown in Table 2. It should be noted that Table 2 shows the OLS estimates under robustness regression conditions, providing the impact of government subsidies on enterprise innovative performance. By controlling the scale, Age of enterprise, R&D investment, ownership type, export, etc., we can find that total government subsidy significantly and positively affected the innovation performance of enterprises at the confidence level of 1%. After substituting whether to enjoy government subsidies into the OLS regression equation for the robustness of results, it can be seen that government subsidies still significantly affected the innovative performance of enterprises. Therefore, it can be said that government subsidies can positively affect the innovation performance of enterprises. Therefore, is the enterprise innovation promoted by government subsidies an imitative innovation or an independent innovation? This paper will make a detailed analysis in the following section.

**Table 2:** Impact of government subsidies on enterprise innovative performance.

**Variable name**	**Explained variable (Logarithm of new product sales in 2015)**			
	**(1)**	**(2)**	**(3)**	**(4)**
Total government subsidies	0.651^***^ (0.0933)	0.219^**^ (0.104)		
Whether to enjoy government subsidies			2.380^***^ (0.364)	0.853^**^ (0.363)
R&D investment		0.549^***^ (0.0646)		0.550^***^ (0.0633)
Age of enterprise		−0.380^*^ (0.230)		−0.367 (0.229)
Scale		0.328 (0.269)		0.407 (0.266)
Export or not		0.349 (0.342)		0.342 (0.341)
Education level of top leaders		0.924^**^ (0.442)		0.904^**^ (0.433)
State-owned enterprises		−0.252 (0.484)		−0.253 (0.485)
Foreign enterprises in Hong Kong, Macao and Taiwan		−1.398^***^ (0.443)		−1.421^***^ (0.448)
Foreign enterprises in non-Hong Kong, Macao and Taiwan		−1.198^*^ (0.706)		−1.270^*^ (0.705)
Fixed effect of region	Yes	Yes	Yes	Yes
Fixed effect of industry	Yes	Yes	Yes	Yes
Sample amount	676	676	676	676
R-squared	0.219	0.372	0.204	0.372

(1) The above results were calculated by stata14.0; (2) The figures in brackets were Robust Std. Error; (3)

* was the significance level of 10%,

** was the significance level of 5%, and

*** was the significance level of 1%.

### Government subsidies, independent innovation and imitative innovation

Therefore, does the enterprise innovation performance promoted by government subsidies belong to independent innovation? If not, is it an “imitative innovation”? This paper selected the total number of patents granted and the number of domestic and foreign patents granted to analyze the “independent innovation.” Furthermore, this paper sets the total number of patents introduced and the number of domestic and foreign patents introduced to analyze the “imitative innovation.” The empirical results are shown in Tables 3, 4.

**Table 3:** Government subsidies and enterprise “independent innovation.”

**Variable name**	**Explained variable (Logarithm of new product sales in 2015)**		
	**(1)**	**(2)**	**(3)**
Total government subsidies	0.308^**^ (0.143)	0.305^**^ (0.144)	0.263^**^ (0.113)
Total government subsidies * Total number of patents granted	-0.0769^*^(0.0429)		
Total number of patents granted	0.690^***^ (0.219)		
Total government subsidies ^*^ Number of domestic patents granted		-0.0785^*^(0.0442)	
Number of domestic patents granted		0.719^***^ (0.223)	
Total government subsidies ^*^ Number of foreign patents granted			**-0.0872 (0.0642)**
Number of foreign patents granted			0.558 (0.480)
R&D investment	0.418^***^ (0.0744)	0.413^***^ (0.0748)	0.539^***^ (0.0649)
Age of enterprise	−0.403^*^ (0.230)	−0.401^*^ (0.230)	−0.362 (0.230)
Scale	0.257 (0.280)	0.251 (0.280)	0.272 (0.279)
Export or not	0.279 (0.346)	0.284 (0.346)	0.345 (0.350)
Education level of top leaders	0.810^*^ (0.430)	0.812^*^ (0.429)	0.861^**^ (0.438)
State-owned enterprises	−0.123 (0.464)	−0.116 (0.464)	−0.167 (0.477)
Foreign enterprises in Hong Kong, Macao and Taiwan	−1.401^***^ (0.443)	−1.406^***^ (0.443)	−1.432^***^ (0.449)
Foreign enterprises in non-Hong Kong, Macao and Taiwan	−0.742 (0.749)	−0.719 (0.745)	−0.833 (0.747)
Fixed effect of region	Yes	Yes	Yes
Fixed effect of industry	Yes	Yes	Yes
Sample amount	655	655	655
R-squared	0.387	0.388	0.376

(1) The above results were calculated by stata14.0; (2) The figures in brackets were Robust Std. Error; (3)

* was the significance level of 10%,

** was the significance level of 5%, and

*** was the significance level of 1%.

**Table 4:** Government subsidies and enterprises “imitative innovation.”

**Variable name**	**Explained variable (Logarithm of new product sales in 2015)**		
	**(1)**	**(2)**	**(3)**
Total government subsidies	0.184^**^ (0.0833)	0.210^*^ (0.111)	0.214^**^ (0.108)
Total government subsidies ^*^ Total number of patents introduced	0.352^*^(0.211)		
Total number of patents introduced	−0.919^**^ (0.455)		
Total government subsidies ^*^ Number of domestic patents introduced		**0.0669 (0.0971)**	
Number of domestic patents introduced		−0.829^*^ (0.499)	
Total government subsidies ^*^ Number of foreign patents introduced			0.415^**^(0.162)
Number of foreign patents introduced			−1.547^*^ (0.893)
R&D investment	0.597^***^ (0.0522)	0.566^***^ (0.0647)	0.556^***^ (0.0642)
Age of enterprise	−0.357 (0.217)	−0.427^*^ (0.233)	−0.392^*^ (0.230)
Scale	0.205 (0.224)	0.341 (0.273)	0.278 (0.267)
Export or not	0.287 (0.296)	0.294 (0.342)	0.317 (0.342)
Education level of top leaders	0.576 (0.489)	0.842^*^ (0.436)	0.848^*^ (0.435)
State-owned enterprises	−0.289 (0.433)	−0.347 (0.482)	−0.348 (0.489)
Foreign enterprises in Hong Kong, Macao and Taiwan	−1.227^***^ (0.431)	−1.433^***^ (0.451)	−1.406^***^ (0.451)
Foreign enterprises in non-Hong Kong, Macao and Taiwan	−0.990^*^ (0.524)	−1.273^*^ (0.692)	−1.176^*^ (0.698)
Fixed effect of region	Yes	Yes	Yes
Fixed effect of industry	Yes	Yes	Yes
Sample amount	671	671	671
R-squared	0.333	0.376	0.375

(1) The above results were calculated by stata14.0; (2) The figures in brackets were Robust Std. Error; (3)

* was the significance level of 10%,

** was the significance level of 5%, and

*** was the significance level of 1%.

First, this paper placed the interactive item between the total number of patents granted and the government subsidies into the model. The results are shown in Table 3. According to the empirical results, the interactive item was significantly negative, indicating that government subsidies and independent enterprise innovation can curb the innovation performance of enterprises. The greater the government subsidies, the more significant their direct role in promoting enterprises' innovative performance. However, it will indirectly weaken the enterprises' independent innovation in promoting the innovation performance of enterprises. Thus, this paper placed the interactive item between the number of domestic and foreign patents granted into the model. The regression model (2) shows that the interaction between government subsidies and independent innovation was significantly negative. Although the interactive item in the regression model (3) was insignificant, the government subsidies failed to improve the enterprises' R&D ability for new products, not to mention the innovation performance of enterprises. Therefore, the independent innovation mechanism did not play a positive role, and the government subsidies had an extrusion effect on independent innovation used for innovation performance improvement.

Next, this paper analyzes the imitative innovation of enterprises, and the results are shown in Table 4. By substituting the total number of patents introduced into the regression model (1) as the interaction term, we can find that the interactive item between the total number of patents introduced and the government subsidies was significantly positive, which suggests that government subsidies can improve the innovation performance of enterprises by stimulating enterprises to introduce more domestic and foreign patents. Government subsidies encourage enterprises to purchase existing technical achievements in the short term to meet the acceptance requirements of government subsidies faster and lay a foundation for future government subsidies.

Then, the number of introduced domestic and foreign patents was placed into the regression model as the “imitative innovation” indicator. The results were consistent with the total number of patents introduced. Although the interactive item coefficient between the number of domestic patents introduced and the government subsidies was not significant, it was positive; the interactive item coefficient between the number of foreign patents introduced and the government subsidies was positive and significant. Under the premise of fully controlling the factors, like enterprise, industry, region, scale, Age of enterprise, R&D investment and ownership type, export or not, government subsidies stimulated enterprises to make the “imitative innovation” and buy domestic and foreign patents to improve the innovation performance of enterprises. The government subsidies stimulated enterprises to form imitative innovation.

This paper also classified the government subsidies to grasp the heterogeneity effect of different government subsidies on enterprise imitative innovation. The empirical results are shown in Table 5. This paper further put the interactive item between the innovation-related government subsidies, such as environmental subsidies, high-tech subsidies and technical innovation funds and the enterprise imitative innovation variable into the regression model. The results showed that the interactive item between the two types of government subsidies of high-tech subsidies and technical renovation funds and the imitative enterprise innovation was significantly and positively related, which meant that the two types of government subsidies were key for enterprises to form imitative innovation. While the interactive item between the environmental subsidies and the enterprise imitative innovation was significantly negative, which indicated that the ecological subsidies could not make enterprises adopt imitative innovation. The reason may be that there were clear rigid requirements for equipment purchase and emission reduction in terms of the environmental subsidies for enterprises, and enterprises failed to satisfy the needs through the introduction or purchase of patents, so they did not promote enterprises to have imitative innovation.

**Table 5:** Government subsidies and enterprises “imitative innovation.”

**Names of variables**	**Explained variable (log value of new product sales in 2015)**		
	**Model 1**	**Model 2**	**Model 3**
Environmental subsidies	−0.0926 (0.218)		
Environmental subsidies * Total number of patents introduced	-1.904^***^(0.484)		
High-tech subsidies		0.844^***^ (0.151)	
High-tech subsidies ^*^ Total number of patents introduced		1.012^**^(0.481)	
Technical innovation funds			0.0693 (0.200)
Technical innovation funds ^*^ Total number of patents introduced			2.743^***^(0.538)
Total number of patents introduced	0.611^***^ (0.0636)	0.554^***^ (0.0644)	0.613^***^ (0.0643)
R&D investment	0.261 (0.494)	0.180 (0.538)	−0.108 (0.498)
Age of enterprise	0.0678 (0.213)	−0.0406 (0.211)	0.0266 (0.214)
Scale	1.045^***^ (0.258)	0.868^***^ (0.257)	1.010^***^ (0.255)
Export or not	1.188^***^ (0.322)	1.097^***^ (0.318)	1.191^***^ (0.323)
Education level of top leader	1.932^***^ (0.473)	1.673^***^ (0.464)	1.903^***^ (0.472)
State-owned enterprises	−0.227 (0.467)	−0.272 (0.444)	−0.165 (0.465)
Foreign enterprises in Hong Kong, Macao and Taiwan	−1.584^***^ (0.450)	−1.455^***^ (0.430)	−1.557^***^ (0.449)
Foreign enterprises in non-Hong Kong, Macao and Taiwan	−0.850 (0.602)	−0.823 (0.598)	−0.894 (0.602)
Fixed effect of region	Yes	Yes	Yes
Fixed effect of industry	Yes	Yes	Yes
Sample amount	809	809	809
R-squared	0.177	0.213	0.176

(1) The above results were calculated by stata14.0; (2) The figures in brackets were Robust Std. Error; (3)

* was the significance level of 10%,

** was the significance level of 5%, and

*** was the significance level of 1%.

## Conclusions and policy suggestions

Under the premise of fully controlling the enterprise, industry, region and time effect, an econometric test on large samples for the internal reasons behind imitative innovation of Chinese enterprises has been conducted by analyzing the data of government subsidies. By reviewing the previous literature, we analyzed the reasons behind the imitative innovation of enterprises, including enterprises' rational choice of cost-gain, property rights system, human capital, and policy environment, but all these methods failed fundamentally explain the change of enterprise innovation behaviors, especially the change in enterprise innovation mode selection. According to this paper, government subsidies, which were key to the formation of imitative innovation, stimulated enterprises to form imitative innovation. Through empirical research, we found that government subsidies stimulated enterprises to make “imitative innovation” through patent purchase rather than independent R&D. Government subsidies were used for low-risk “imitative innovation” because of enterprises' rent-seeking behavior and low R&D ability and the review of government subsidy projects.

### Policy recommendation

Based on the above empirical research results, this paper puts forward the following policy recommendations:

First, it is recommended that the government reduce or withdraw from its intervention in the highly risky field of enterprise innovation. According to the analysis results, government subsidies fail to stimulate the enterprises' abilities for independent innovation because enterprises are inclined to adopt the low-risk innovation form of “imitative innovation” when improving innovation levels. Based on this, government subsidies have only helped improve enterprises' innovation ability superficially, but the independent innovation ability of enterprises has not been fundamentally improved. Therefore, the government should reduce or withdraw from its intervention in fiscal policy and suspend other policies in the high-risk field of enterprise innovation. When it comes to large enterprises, the government may procure their specific products to expand the market demand for relevant industries and thus promote the independent innovation of the industries. For small and medium-sized enterprises, the government can provide more supportive policies through preferential policies, such as tax reduction and tax return, as most of these enterprises are still in the initial stage of enterprise of independent R&D.

Secondly, innovative subsidies' achievement inspection and acceptance mechanism should be reformed. In order to prevent enterprises from using subsidy funds for imitative innovation, the government can change the prior subsidy into post-subsidy and conduct strict inspection and acceptance of the subsidy results. In addition, the targeted enterprises for acceptance should be classified, enterprises with strong independent innovation ability should be strictly audited, and small and medium-sized enterprises with poor autonomy should be provided more time for independent innovation by appropriately expanding the audit period.

Thirdly, the achievement evaluation mechanism for innovative subsidies needs to be established. In addition to accepting the number of patents, an innovative performance evaluation system needs to be established to review the independent R&D expenditure and the number of patents for independent application and strictly regulate the audit by purchase.

### Limitations and future research

First, the scope of the research is limited to a particular emerging economy (China). China's institutions, culture, and so on may be different from those of other economies, although China has the largest emerging economy. Because of this, the selection of alternative economies or industries may have an impact on the findings of the research. The objects of the research can be chosen again for use as test subjects in subsequent studies. Second, to supplement the findings of previous research, we can conduct additional research in the future to investigate the influence of other internal factors of the enterprise, such as the type of enterprise ownership and the degree to which the enterprise is financially standardized. Finally, regarding the influence of the enterprise's surrounding environment on its operations, our investigation considers only the institutional setting of the innovation subsidy. It is necessary to conduct additional research in order to investigate the effects of other policies (such as high-tech enterprise qualification recognition, talent subsidy, and so on), as well as the effects of different external environments (such as the market environment).

## Data availability statement

The original contributions presented in the study are included in the article/supplementary material, further inquiries can be directed to the corresponding author/s.

## Author contributions

FS and CZ: statistical data analyses and writing of the manuscript. Both authors contributed to the article and approved the submitted version.

## Funding

This work was supported by “the Fundamental Research Funds for the Central Universities” (No. 21lzujbkydx029); the MOE Layout Foundation of Humanities and Social Sciences (No. 20YJA790045); Key Projects of Philosophy and Social Sciences Research, Ministry of Education (No. 15JZD024).

## Conflict of interest

The authors declare that the research was conducted without any commercial or financial relationships construed as a potential conflict of interest.

## Publisher's note

All claims expressed in this article are solely those of the authors and do not necessarily represent those of their affiliated organizations, or those of the publisher, the editors and the reviewers. Any product that may be evaluated in this article, or claim that may be made by its manufacturer, is not guaranteed or endorsed by the publisher.
